# Mo-Si-B Alloy Formed by Optional Laser Melting Process

**DOI:** 10.1155/2022/4996265

**Published:** 2022-06-23

**Authors:** Zhengyou Guo, Renheng Han, Yanan Li, Yanqing Zhu, Bin Zhang, Hexin Zhang

**Affiliations:** ^1^College of Materials Science and Chemical Engineering, Harbin Engineering University, Harbin, Heilongjiang 150001, China; ^2^Key Laboratory of Superlight Materials and Surface Technology, Ministry of Education, Harbin Engineering University, Harbin, Heilongjiang 150001, China

## Abstract

In this research article, the molybdenum alloy was prepared by solid-solid doping, selecting pure Mo powder, amorphous Si powder, and B powder as the experimental raw materials for SLM molding. The density and mechanical properties of Mo-Si-B alloys prepared by SLM technology under different processes and compositions were explored, and at the same time, the microstructure of the obtained alloy was observed. The result shows that, with a laser power of 250 W, a scanning speed of 500 mm/s, and a scanning distance of 60 *μ*m, the Mo4.5-Si2-B (at.%) alloy has the highest forming rate under the 120°parameters of the rotating scanning strategy, and the highest density is 94.22%.

## 1. Introduction

At the same time, the resource reserves of molybdenum metal in China are also extremely rich, accounting for 50% of the world's molybdenum resources, ranking first in the world. Selective laser melting (SLM) is a type of metal additive manufacturing (AM) technology, and it is an emerging advanced material manufacturing technology in recent years [1, 2]. This technology has the characteristics of high degree of flexibility in the manufacturing process, excellent mechanical and chemical properties of the manufactured parts, and small influence on the difficulty of processing by the size and complexity of the product [3]. Because of its controllable forming atmosphere and one-time forming of complex structures [4], this makes it a forward-looking new manufacturing method for the manufacture of molybdenum-based super alloy parts. Mo-Si-B series alloys were initially studied in depth on the basis of molybdenum silicide high-temperature structural materials; now, because of its more comprehensive performance such as high melting point (melting point greater than 2000°C), excellent high temperature strength, creep resistance, and excellent oxidation resistance [5] having attracted much attention, it has broad application prospects in aerospace and other fields and has also received more attention from many scholars in recent years.

At present, in the research of relative density of SLM forming metal, the scholar Wang Huiyang used the MCP Realizer250 SLM equipment to study the formation of stainless steel [6]. It is found that the high laser power, low scanning density, and increasing energy density can easily increase the density of the molded part; scholars such as Zhang Yangjun used the self-developed SLM equipment formation to study the relative density of Ti powder SLM forming, prepared pure titanium parts with a relative density of 96%, and discussed the influence of laser power and scanning speed on relative density [7]; Lin Xin used spheroidized loose molybdenum powder as raw material, a pure molybdenum sample without cracks was prepared by the selective laser melting method, and it is found that the spheroidization of the precursor powder can increase its density [8]. Among them, Meier H [9] studied the laser power, scanning speed, and other parameters of the SLM process according to the high temperature resistance characteristics of molybdenum powder; the investigation found that the use of high laser power and low layer thickness density can improve the compactness of the molded parts. However, there are still relatively few related studies in the field of SLM forming Mo-Si-B alloys, and there is no in-depth exploration of the mechanical properties of the materials after forming.

Mo-Si-B alloys with different compositions are prepared by selective laser melting technology, exploring the optimal process parameters in the printing process and considering the material forming rate and density; the selected parameters are laser power, 250 W; scanning speed, 500 mm/s; and scanning strategy, 120°offset rotation as the optimal printing parameter combination; under this parameter, the material forming rate reaches 100%; and the maximum density is 94.22%.

## 2. Test Materials and Methods

In this experiment, a solid-solid doping method was used to design and prepare three different molybdenum alloys, the outstanding advantages are that the operation is convenient, the synthesis process is simple, the particle size is uniform, the force is controllable, and the pollution is less, and at the same time, the hard agglomeration phenomenon that is easy to occur in the liquid phase can be avoided or reduced, the cost is low and choose 300 mesh, pure Mo powder with a particle size of 13–53 *μ*m and 500 mesh, and amorphous Si powder and B powder with a particle size of 2–25 *μ*m are used as raw materials for selective laser melting molding. The powder morphology shown in Figures 1(a) and 1(b) is the SLM-formed pure Mo powder and the high-magnification scan of Mo powder, respectively. Figures 1(c) and 1(d) show the mixed powder. At all laser powers, the relative density values decreased in the higher scan speed range (400 to 1200 mm/s).

This experiment is based on different atomic composition ratios, three Mo-Si-B alloys with different composition are designed respectively, and the specific composition is shown in Table 1:

The model of the experimental equipment selected is FS721M molding equipment, and the parameters of the equipment are shown in Table 2:

This experiment uses the ICP-AES method to determine the element content in the printed sample [10]; for different printing process parameters, the size of the printed sample is selected as 10 × 10 × 5 mm; the room temperature toughness of the printed sample was measured by a three-point bending test with a sample size of 60 × 10 × 10 mm. Definition: the theoretical density of different Mo-Si-B alloys is jointly calculated by the weight percentages of the respective components, using Archimedes drainage method to measure the actual density of printed samples with different components and different process parameters; the heat treatment process is expected to eliminate the cold cracks and internal stress of the Mo-Si-B alloy after laser melting in the selected area, the specific heat treatment method is to use sandpaper or electric grinder to polish the surface of the sample to remove the attached particles, and then encapsulate the sample in a ceramic tube filled with inert gas, the packaged sample will be placed in a heat treatment furnace at a temperature of 1200°C and take it out after keeping it evenly for 24 h, that is, the heat treatment process is completed.

## 3. Test Results and Analysis

### 3.1. The Influence of SLM Process Parameters on the Forming Rate and Microstructure of Mo-Si-B Alloy

Design five sets of parameters for 1-1 combination, numbered 1–5 respectively, the specific parameters of the process and the corresponding material forming rate under each process are shown in Table 3:

Analysis of Table 3 can be obtained with the increase of printing power and scanning speed, the forming rate shows a trend of rising first and then falling, among them [11]. The forming rate of the two sets of parameters numbered 3 and 4 dropped sharply; on the whole, the laser power is 250 w; when the scanning speed is 500 mm/s, the material forming rate is the highest, reaching 100%.

After the material is formed, the density and the number and distribution of defects are also one of the important evaluation criteria, density is negatively correlated with internal void defects, that is to say [12], the sample with fewer holes and defects is macroscopically dense. The specific density is shown in Figure 2.

It can be seen from Figure 2 that the density generally increases with the increase of the volume energy density, the high volume energy density has an obvious effect on eliminating holes and incomplete melting defects, the highest density can reach 94.22%, and the performance of density is related to holes. Hot cracks during the forming process can also cause fluctuations in the density performance [13].

Observe the micromorphology of sample 1-1 under different printing powers, and compare the distribution of cracks and holes as shown in Figure 3.

Based on the schematic diagram of the microscopic morphology, we have obtained the reason for the change in density: (a) the pores are densely distributed, and the density performance is the worst. As the volumetric energy density increases, the number and size of the holes decrease; as a result, the density gradually increases; on the other hand, the number and size of cracks are gradually expanding, in (e), it is obvious that the thermal cracks spread to a staggered distribution on the surface [14]. Thermal cracks are mostly along the crystal cracks, mainly appearing at the grain boundary with more impurities, and obvious oxidation color appears on the crack section, in the SLM forming process, due to the repeated thermal influence process, the size of the thermal cracks will expand and extend.

Combined with the above experimental results, comprehensive consideration of forming rate and density selected relatively optimal process parameters such as the laser power is 250 W, the scanning speed is 500 mm/s, and the scanning strategy is 120°offset rotation.

### 3.2. Density and Mechanical Properties of Mo-Si-B Alloys with Different Compositions under Optimal Process Parameters

#### 3.2.1. Density

First, calculate and compare the density under different components to analyze its actual forming quality. The element content measured by the ICP-AES method is shown in Table 4 and Figure 4.

Figure 4 shows the density of different alloy components after forming under selected process parameters and the theoretical density of the composition. It can be seen from the figure that when the content of alloying elements is small, it has the highest density; as the content of alloying elements increases [15], the density shows a significant downward trend. The two reasons for the decline are the increase in the B element content in the raw materials; in the actual forming process, the B element content is greatly burned, and the density is not as expected. On the other hand, after the element changes, the processing parameters are no longer applicable, resulting in an increase in the number of defects in the molding process.

#### 3.2.2. Bending Strength

Pure molybdenum metal is a completely brittle material at room temperature, the rigidity is extremely high, and it can obtain great toughness after forming a solid solution with the alloying elements Si and B. However, the intermetallic compounds formed after solid solution are also rigid materials with high strength and low toughness [16]. As can be seen from Figure 5(a), the maximum bending stress is when the alloy composition is Mo-4.5Si-2B, the bending stress is 978.6 N. As the content of alloying elements increases, the maximum bending force decreases, which is not consistent with the actual phase composition performance obtained; from the previous density situation, it should be the existence of defects that drag down the performance.

We expect to achieve the purpose by eliminating cold cracks and improving performance through heat treatment. However, from Figure 5(b), the bending strength of the samples before and after the heat treatment was compared, and the bending strength is shown in Table 5.

Before and after heat treatment, in addition to the increase in strength of Mo-4.5Si-3.5B, the strength of the other samples has decreased, but Mo-4.5Si-3.5B showed obvious brittle fracture after heat treatment. The increase in strength and the decrease in ductility should come from the increase in the content of intermetallic compounds, improving the strength of the bending force and reducing its ductility.

From the results of the three-point bending experiment, the addition of Si and B elements produces a certain degree of plasticity, and plastic performance mainly comes from *α*-Mo solid solution. When the solid solution content is exceeded, the Si and B elements will damage the performance. The results showed that the heat treatment process tried to eliminate internal stress and reduce cold cracks but failed to achieve [17].

#### 3.2.3. Brittle Toughness

The fracture toughness is used to measure the toughness performance of each component and the samples before and after heat treatment. The experimentally measured fracture toughness Kq is shown in Table 6 and compared with another molybdenum-based alloy using the same test method. As can be seen from the table, the fracture toughness of the molybdenum-based alloy processed by SLM is much lower than that of other *α*-Mo with high volume fraction, hot cracks and hole defects during SLM processing greatly affect the fracture toughness. The performance difference between the components is also affected by defects and cannot be accurately distinguished, but overall, it still shows that it has not been heat-treated. As the content of Si and B elements increases, the fracture toughness will decrease. This is consistent with the phase composition, and after the heat treatment, the internal stress drops, and the coarsening of crystal grains leads to a decrease in toughness as a whole [18, 19].

The microscopic morphology of the fracture after bending and fracture is shown in Figure 6. It can be seen from Figure 6(a) that the main form of the fracture is a quasicleavage fracture, and the obvious river pattern can be seen in the lower left corner; in the form of cleavage fracture, there are obvious dimples in the enlarged area, at the same time, in (a), there are obvious bifurcation and cracking characteristics, which are consistent with the crack characteristics in the stress corrosion fracture. In Figure 6(b), there are also pits that appear when the particles are pulled out, and there are also particles that still remain spherical. The particles are in good melting condition but still maintain the circular boundary, and the crack propagation also proceeds along the spherical boundary, in Figure 6(c). There is an obvious incomplete melting phenomenon; therefore, the samples before heat treatment can be considered to have a small amount of plasticity and toughness. This is also the reason why there is no direct stress unloading in the bending test, and the rapid decline in performance in Mo-5Si-5B can be attributed to poor density performance. At the same time, the samples after heat treatment are concentrated in brittle fracture, and almost all of the steps in Figure 6(d) are cleavage and fracture steps. However, the characteristics of quasicleavage fractures such as Lailai Ridge are less. In Figure 6(e), there are also a large number of dissociated surfaces and river-like patterns, ad this is also consistent with the stress unloading that occurs during the bending process. In the Figure 6(f), affected by heat treatment, internal defects may be reduced to a certain extent; therefore, the toughness performance is improved compared with other samples [20].

### 3.3. Analysis of the Heat Treatment Process

#### 3.3.1. Before Heat Treatment

When the alloy composition is the same, the inside of the formed sample contains obvious different phases, especially when Mo-5Si-5B is the most obvious, and the microstructure of the three components was further observed by SEM. The organization is shown in Figures 7(a)–7(c):

(a) is mainly *α*-Mo, the grain size is not uniform, and the distribution pages are extremely uneven, and the grain distribution in (b) is the same as in (a) and (c). There are more second phases in the middle, it can be clearly observed from the scan image that there is a clear second phase at the grain boundary, and the second phase isolates *α*-Mo into a discontinuous state. Discontinuous *α*-Mo is compared to continuous *α*-Mo, and plastic toughness performance will have a significant decline [21]. At the same time, the second phase in Mo is mostly brittle. After being subjected to a force exceeding its maximum strength, damage will occur, this can also explain the worst plastic toughness performance of Mo-5Si-5B in the three-point bending experiment [22].

#### 3.3.2. After Heat Treatment

From the perspective of mechanical tests, the performance after heat treatment has been reduced, did not achieve the purpose of trying to eliminate cold cracks and improve performance before treatment, and further observe the structure of the heat-treated sample. The heat treatment organization is shown in Figures 8(a) and 8(b).

In Figure 8(a) There is no obvious change in the morphology of the middle structure, and some grains are coarsened. However, there are still a large number of fine crystals. In Figure 8(b) When the alloy composition content increases, there is a needle-like second phase dispersion distribution. When the element content further rises, a large number of dendrites in Figure 8(c) will appear in some areas, the appearance of dendrites is the result of further increase in element content, connected by the needle-like second phase to form dendrites. The appearance of dendrites has a weakening effect on performance [23, 24]. At the same time, the heat treatment process of molybdenum-based alloys is also accompanied by embrittlement caused by grain coarsening. Therefore, the two effects make the performance of the alloys of each component have different degrees of decline after heat treatment. The microstructure of the SLM-formed CoCrMo alloy was observed, and the relevant components were tested. The molded part mainly has one phase at room temperature, the microstructure is dense, and the melt channel characteristics are obvious.

## 4. Conclusion

The purpose of using additive manufacturing technology to process molybdenum-based superalloys is to explore the feasibility of using direct forming technology in refractory alloys, the influence of trace alloying elements Si and B on the properties and microstructure of Mo-based alloys formed by SLM, as well as the related mechanism of the heat treatment process affecting the mechanical properties of materials. The following conclusions are obtained:

1. Choose a Mo-Si-B alloy whose atomic composition (at.%) is Mo (93.5), Si (4.5), and B (2), given multiple sets of laser melting process parameters for selected areas for printing, comprehensive consideration of forming rate and density, and selected relatively optimal process parameters such as laser power, 250 W; scanning speed, 500 mm/s; and scanning strategy, 120° offset rotation. Under this parameter, the forming rate reaches 100%, and the highest density reaches 94.22%.
2. Through the three-point bending experiment, it is found that the addition of Si and B elements adds some plasticity to the material, and the maximum bending force is 978.6 N when the composition is Mo-4.5Si-2B before heat treatment.
3. Observing the microstructure of different compositions, the microscopic difference of different structures without heat treatment is not big. When the alloy composition content is high, the second phase appears at the grain boundary. After heat treatment, as the alloy composition content increases, obvious second phase precipitation appears. Mo-4.5Si-3.5B isneedle-like, and Mo-5Si-5B is dendritic. Because the heat treatment is heated for a long time, the carbon and other alloying elements in it can be fully diffused, mainly to make it uniform, so that, after the material becomes uniform, its properties such as tensile strength and toughness will be greatly improved. Experiments have confirmed the weakening of the performance during the heat treatment process, and the mechanism of the weakening has been given.

## Figures and Tables

**Figure 1:** The morphology of powder and mixed powder.

**Figure 2:** Schematic diagram of relative density and density evolution of sample numbers under different printing powers.

**Figure 3:** Schematic diagram of the micromorphology of 1-1 under different printing powers: (a) parameter combination 1, (b) parameter combination 2, (c) parameter combination 3, (d) parameter combination 4, and (e) parameter combination 5.

**Figure 4:** Density under different ingredients.

**Figure 5:** Three-point bending test of samples with different compositions ((a) without treatment and (b) after heat treatment).

**Figure 6:** Fracture before heat treatment: (a) Mo-4.5Si-2B and (b) Mo-4.5Si-3.5 B. After heat treatment: (c) Mo-5Si-5B, (d) Mo-4.5Si-2B, (e) Mo-4.5Si-3.5 B, and (f) Mo-5Si-5B.

**Figure 7:** The microstructure of different compositions (a) Mo-4.5Si-2B, (b) Mo-4.5Si-3.5 B, and (c) Mo-5Si-5B.

**Figure 8:** Metallographic structure of different compositions after heat treatment. (a) Mo-4.5Si-2B, (b) Mo-4.5Si-3.5B, (c, d): Mo-5Si-5B).

**Table 1:** Material design composition.

Element	Element (at. %)		
	1-1	1-2	1-3
Mo	93.5	92	90
Si	4.5	4.5	5
B	2	3.5	5

The three selected Mo-Si-B alloys are as follows: 1-1, Mo (93.5) Si (4.5) B (2); 1-2, Mo (92) Si (4.5) B (3.5); and 1-3 Mo (90) Si (5) B (5).

**Table 2:** Printing equipment performance parameters.

Technical parameter	FS721M
Forming cylinder size (L × W × H)	720 × 420 × 420 mm
Thickness of powderlayer	0.02∼0.1 mm (adjustable)
Scan speed	10 m/s (highest)
Laser system	Fiber laser and dual laser (2 ^*∗*^ 500 W)
	Four lasers (4 × 500 W)
Spot size	Profile scan diameter, 70 *μ*m
	Fill scan diameter, 70∼200 *μ*m

**Table 3:** Combination forming rate of different parameters.

Parameter			Forming rate (%)
Serial number	Laser power (W)	Scan speed (mm/s)	
1	250	400	80
2	250	500	100
3	300	500	80
4	300	400	40
5	325	400	20

**Table 4:** Molybdenum silicon boron element content and theoretical density after ICP measurement.

Serial number	Mo (at. %)	Si (at. %)	B (at. %)	Theoretical density (kg/m^3^)
1	94.9910	4.4910	0.5179	9805.920183
2	94.5278	4.5577	0.9144	9769.623809
3	93.8825	4.7564	1.3611	9719.016331

**Table 5:** Test sample bending strength under different components and processes.

Element	Section factor (mm^3^)	Maximum bending force, 10^3^ (N)	Bending strength, MPa
Mo-4.5Si-2B	210.33	0.9786	46.53
Mo-4.5Si-3.5B	206.43	0.7575	36.70
Mo-5Si-5B	172.21	0.7573	24.57
Mo-4.5Si-2B (heat treatment)	204.16	0.9341	45.75
Mo-4.5Si-3.5B (heat treatment)	201.45	1.3490	31.46
Mo-5Si-5B (heat treatment)	186.49	0.7573	40.61

**Table 6:** Fracture toughness of samples with different compositions.

Sample		Cross-sectional area, mm^2^	Absorbtion energy, mJ	Fracture toughness, kq, $\text{MPa}\sqrt{m}$
Element	Processing			
Mo-4.5Si-2B	Without	7044.16	177.23	2.94
Mo-4.5Si-3.5B		6899.63	201.31	3.16
Mo-5Si-5B		6262.10	43.30	1.54

Mo-4.5Si-2B	Heat treatment	7002.42	93.49	2.14
Mo-4.5Si-3.5B		6930.97	109.97	2.33
Mo-5Si-5B		6429.45	96.86	2.27
Mo-12Si-8.5B-1Zr				12.4
Mo-12Si-8.5B				9.0

## Data Availability

The data used to support the findings of this study are available from the corresponding author upon request.
